# RNF181 modulates Hippo signaling and triple negative breast cancer progression

**DOI:** 10.1186/s12935-020-01397-3

**Published:** 2020-07-06

**Authors:** Rui Zhou, Yinlu Ding, Min Xue, Bin Xiong, Ting Zhuang

**Affiliations:** 1 Department of Thyroid and Breast Surgery, Zhongnan Hospital of Wuhan University, Wuhan, China; 2 Hubei Cancer Clinical Study Center, Hubei Key Laboratory of Tumor Biological Behaviors, Wuhan, Hubei 430071 People’s Republic of China; 3 Department of General Surgery, The Second Hospital, Cheeloo College of Medicine, Shandong University, Jinan, Shandong People’s Republic of China; 4 Henan Key Laboratory of Immunology and Targeted Therapy, School of Laboratory Medicine, Henan Collaborative Innovation Center of Molecular Diagnosis and Laboratory Medicine, Xinxiang Medical University, Xinxiang, 453003 Henan People’s Republic of China; 5 Department of Gastrointestinal Surgery, Zhongnan Hospital of Wuhan University, Wuhan, China

**Keywords:** RNF181, Hippo, YAP, TNBC, Ubiquitin

## Abstract

**Background:**

Breast cancer ranks No. 1 in women cancer incidence, while triple negative breast cancer (TNBC) is the most aggressive and the worst prognostic subtype in all breast cancer subtypes. Compared with estrogen receptor alpha positive breast cancer, which could be well controlled by endocrine therapy, TNBC is lack of mature molecular targets for medical therapy. Thus, it is urgent and necessary to discovery the carcinogenic mechanism and potential therapeutic targets for TNBC. Recent studies reveal that Hippo/YAP signaling is an important mediator for TNBC progression. Our current study investigates the role of RING finger protein RNF181 in modulation Hippo/YAP signaling.

**Methods:**

YAP and RN181 protein level were measured by western blot, while the Hippo classical target genes were measured by real-time PCR. WST1 assay were used to measure cell proliferation, the trans-well and wound healing were used to measure the cell migration and invasion capacity. Protein stability and ubiquitin assay were used to detect the YAP protein ubiquitin and stability. The immuno-precipitation assays were used to detect the protein interactions. Immuno-staining was used to detect the protein localization of YAP and RNF181, while the ubiquitin-based immuno-precipitation assays were used to detect the specific ubiquitination manner of YAP.

**Results:**

Our current study identified a novel modulator-RNF181 as a positive mediator for Hippo/YAP signaling activation in TNBC. RNF181 depletion significantly inhibited TNBC cell migration, invasion and proliferation, which effect could be rescued by YAP overexpression. RNF181 depletion decreased YAP protein level and Hippo signaling target genes, such as CTGF and CYR61, in TNBC cell lines. Immuno-precipitation assay showed that RNF181 interact with YAP and promoted YAP stability by inhibition K48-linked poly-ubiquitination of YAP in TNBC cells. Besides, public available data showed that RNF181 is elevated in breast cancer and related to poor prognosis in TNBC patients.

**Conclusion:**

Our study provides evidence to establish a non-proteolytic mechanism in modulating Hippo signaling in breast cancer. RNF181 could be an interesting marker for triple negative breast cancer prognostics and therapeutics.

## Highlights

1. RNF181 facilitates YAP/TEAD axis in triple negative breast cancer.
2. RNF181 promotes triple negative breast cancer progression via Hippo signaling.
3. RNF181 controls Hippo signaling in triple negative breast cancer via modulating YAP stability and ubiquitination level.

## Background

Triple negative breast cancer (TNBC) is an aggressive subtype breast cancer, which is lack of expression of estrogen receptor alpha, progesterone receptor and HER2 [1]. TNBC is lack of approved target therapies, which remain a major hindrance for the survival improvement [2]. In addition, TNBC has higher trend to metastasize and poorer overall survival compared with other breast cancer subtypes [3]. Since it is lack of therapeutic targets in TNBC, it is urgent to uncover the oncogenic mechanism and novel targeted therapies for TNBC patients.

The organ hemostasis is dependent on an internal balance among proliferation, apoptosis, stem cell self-renewal and differentiation [4]. These processes are necessary for the tissue hemostasis, while the deviation of such regulation leads development failure or carcinogenesis. The Hippo signaling was shown to play important role in organ size control [5]. The core component of Hippo signaling includes MST1/2, LATS1/2, YAP, TAZ and TEADs. When Hippo signaling is activated MST1/2 phosphorylates LATS1/2, which further phosphorylates YAP/TAZ cytoplasmic retention and degradation. While Hippo signaling is shuttled down, unphosphorylated YAP/TAZ could translocate into the nuclear and associate with several transcriptional factors, including TEADs [6]. Thus, YAP/TAZ are important effectors for Hippo pathway, which could shuttle between cytosol and nuclear.

The abnormality of Hippo signaling could be found in quite a few human cancers [7]. For example YAP gene amplification could be found in live cancer, esophageal cancer and TNBC (https://tcga-data.nci.nih.gov/tcga/). Besides, YAP was shown to be critical in modulating server cancer biological behaviors, including carcinogenesis, cell survival and stem cell maintenance [8]. Depletion YAP or pharmaceutical inhibition YAP could lead to cell death and cell growth inhibition [9, 10]. In breast cancer, population based genomic study showed that Hippo signaling activation was correlated with TNBC breast cancer risk, while high expression of YAP related to poor survival in breast cancer patients [11, 12]. Besides, YAP/TEAD axis was shown to synergize with AP-1 family members in TNBC to promote cancer progression, while depletion of YAP in TNBC cells inhibited migration capacity and proliferation in vitro and in vivo [13]. All these conclusions indicated that Hippo/YAP axis played critical role in TNBC carcinogenesis and progression. Thus targeting YAP protein transactivation could be an appealing strategy for TNBC treatment. However, due to the extensive interaction between YAP and TEAD, directly target YAP-TEAD interaction is still immature in clinics [14]. Our currently study aims to investigate the YAP protein modulators, which could be an alternative strategy for YAP-driven breast cancer.

Ring finger protein 181 (RNF181) belongs to RING finger protein family, and functions as an E3 ubiquitin ligase in regulator multiple cellular processes [15]. For example, RNF181 was shown to bind integrin complex and modulate platelet function in physiological condition [16]. Besides, RNF181 could regulate NFKB signaling via interaction with CARD11 in lymphocytes [17]. However, little is known about RNF181 function in human cancer. Our current study showed RNF181 is an important modulator for Hippo/YAP signaling and in TNBC progression. RNF181 could stabilize YAP protein and inhibit K48 linked poly-ubiquitination, which leads to enhanced YAP target gene expression and cancer progression in TNBC.

## Materials and methods

### RNA extraction and qPCR analysis

Total RNA was used to extract by RNeasy plus mini kits (Tiangen). Real-time PCR was showed as previously described [18]. 36B4 was used for internal reference. The primer sequences were displayed here. RNF181: F: cac aga cga gat aag gct cga a; R: tgg cca ggt ctg tga tca at. 36B4: F: ggc gac ctg gaa gtc caa ct; R: cca tca gca cca cag cct tc. CTGF: F: ctc gcg gct tac cga ctg; R: ggc tct gct tct cta gcc tg. CYR61: F: agc agc ctg aaa aag ggc aa; R: agc ctg tag aag gga aac gc.

### Cell culture

The three species cells include BT549, MDAMB231 and HEK293 cells were used from American Type Culture Collection (ATCC). HEK293 cells were cultured in Dulbecco’s Modified Eagle’s Medium that contains 4,5 g/L glucose and 4 mM l-glutamine (DMEM, 41965, Life Technologies) supplemented with 10% Fetal Bovine Serum (FBS, 10270, Life Technologies). MDAMB231 and BT549 cells grown in RPMI-1640 (42401, Life Technologies) supplemented with 2 mM l-glutamine (25030, Life Technologies) and 10% FBS. All cell lines were subject to cell line authentication. The cell line authentication via Short Tandem Repeat (STR) was performed via PowerPlex 21 system. The STR data of HEK293, MDAMB231 and BT549 cell lines were found consistent with STR data in ATCC.

### Plasmids and siRNA

The Myc-YAP plasmid was acquired by Origene,The Flag-RNF181 plasmid was obtain from Origene. The HA-K48 Ubiquitination plasmids were received from our past study. The Lipofectamin 2000 (1668019, Invitrogen) was used for the plasmids transfection. Small interfering RNAs were used for specific gene knocking-down. The RNF181 siRNA sequences were: CCACUGAUGACGACACUUAdTdT; UAAGUGUCGUCAUCAGUGGdTdT and GAUGCCUUGCCAUCACCUUdTdT; AAGGUGAUGGCAAGGCAUCdTdT. The YAP siRNA sequence were: GCUCAUUCCUCUCCAGCUUTT; AAGCUGGAGAGGAAUGAGCTT. The negative control siRNA sequences were: UUCUCCGAACGUGUCACGUTT; ACGUGACACGUUCGGAGAATT. The RNAiMAX reagent (13778150, invitrogen) was used for siRNA transfection.

### Cell proliferation assay

SiRNF181 or siControl transfect into MDAMB231 and BT549 cells in 24-well plate. Twenty-Four hours after transfection, the cells number was countered and 6000 cells were seeded into 96-well plates. The comparatively cell viability was measured at indicated time points. Cell numbers were determined using the CCK8 cell proliferation reagent as previously described.

### Wound healing assay

BT549 and MDA-MB-231 cells were transfected with 50 µM RNF187 siRNA or sControl. After 24 h, cells were seeded into 6-well plates with 2%FBS. The cells were 100% confluence. The yellow pipette tips were applied for straight scratch. The Cells wound distance was measured every 24 h. The wound healing recovery was expressed as: [1 − (Width of the wound at a given time/width of the wound at t = 0)] × 100%.

### Trans-well assay

The Cell invasiveness was measured using the modified two-chamber plates as before [19]. For invasion assay MDAMB231 cells and BT549 cells were were transfected with 50 μM RNF181 siRNA or sControl. To stimulate invasion, 20% of the serum was added to the 24-well plat by using a serum-free medium in the chamber. After 16 h, cells were carefully removed and the cells that invaded through the membrane were fixed and stained with Crystal Violet Staining solution. The cell numbers are counted by microscope.

### Western blotting

RIPA buffer lysates harvest the cells. Proteins were separated by electrophoresis on SDS-polyacrylamide gel electrophoresis (PAGE) and electro-transferred to PVDF membrane. The antibodies we use include: Anti-RNF181 (SAB1401685, Sigma); Anti-YAP (SC-101199, Santa Cruz); Anti-phospho-YAP (S127) (ab76252, Abcam); Anti-HA (MMS-101R, COVANCE); Anti-myc (9E10, ab9106, Abcam); Anti-GAPDH (GB12002, Servicebio). Membranes were then washed with PBS for three times and incubated with secondary antibodies Peroxidase-Conjugated AffiniPure Goat Anti-Mouse IgG or Goat Anti-Rabbit IgG. Fluorescent signals were visualized with ECL system (GE RRPN 2235).

### Protein stability assays

For BT549 cells were seeded into 24 well-plate and transfected with 50 nM siRNF181 or siControl. After 24 h, cells were treated with 100 µM cycloheximide (C7698, Sigma) for indicated time points. Samples were subject to western blot for YAP degradation.

### Immunofluorescence assay

BT549 cells were fixed with 4% paraformaldehyde in PBS for 10 min, permeabilized with 0.25% Triton X-100 for 5 min, and blocked by 3% BSA in PBS for 1 h. anti-RNF181 polyclonal antibody (SAB1401685, Sigma) and anti-YAP monoclonal antibodies (SC-101199, Santa Cruz) were used, followed by Alexa Flour 647 (Invitrogen) anti-rabbit antibody and FITC-conjugated anti-mouse antibodies (Jackson ImmunoResearch, West Grove, PA). As negative controls, the samples were incubated with the secondary antibodies without primary antibodies. Images were acquired under conditions fulfilling the Nyquist criterion using Nikon A + laser scanning confocal system with a 60X oil NA1.4 objective and pinhole size of 1.0 Airy Unit. The acquired pictures were further processed and assembled using ImageJ.

### Poly-ubiquitination detection assay

To directly detect the enriched K48-ubiquitinated and Myc-YAP from the cell extracts, HEK293T cells were transfected with 0.5 μg K48 Ubi plasmids together with 0.5 μg Flag-RNF181 or Flag-vector. After 48 h, total protein was extracted and pre-cleared with 20 μL protein A (santa cruz, SC-2001) for 2 h. The supernatant was collected and immunoprecipitated by YAP antibody. Western blot with HA antibody was performed to detect K48 poly-ubiquitinated YAP.

### Statistics

Pearson correlation coefficient, Student’s t-test, and Cox regression analysis were applied for comparisons. A P-value of < 0.05 was considered to be statistically significant.

## Results

### RNF181 is higher expressed in breast cancer and correlates with poor survival in TNBC patients

We analyze the public available data of RNF181 in breast cancer database. From the Oncomine database (https://www.oncomine.org), we find that RNF181 is elevated in breast cancer, compared with normal breast tissue in multiple cohorts (Fig. 1a–c). Besides, the KMPLOT database (http://kmplot.com/analysis/) indicates that RNF181 correlate with poor survival in total breast cancer patients and also TNBC patients (Fig. 1d, e). Interestingly, YAP expression shows similar trend in prognosis with RNF181 in TNBC patients (Fig. 1f). Besides, he KMPLOT database (http://kmplot.com/analysis/) indicates that RNF181 correlate with poor survival in TNBC patients in 5 years and 10 years survival (Fig. 1g, h).

**Fig. 1:** RNF181 is elevated in breast cancer samples and correlated with poor prognosis in triple negative breast cancer cells. **a**–**c** RNF181 is increased in mRNA expression in breast cancer samples compared with normal breast tissue from different datasets (https://www.oncomine.org). **d** RNF181 is correlated with poor prognosis in total breast cancer patients (https://kmplot.com). **e** RNF181 is correlated with poor survival in TNBC patients (https://kmplot.com). **f** YAP expression level is correlated with poor survival in TNBC patients (https://kmplot.com). **g** RNF181 is correlated with poor survival in TNBC patients in 5 years follow-up (https://kmplot.com). **h** RNF181 is correlated with poor survival in TNBC patients in 10 years follow-up (https://kmplot.com)

### RNF181 promotes cancer progression and proliferation in TNBC cells

We used BT549 and MDAMB231 cells as representative cell lines for TNBC in most of the experiments. In order to minimize the off-target effects of the siRNAs, two independent siRNAs are used to knock down RNF181. The WST1 assay indicates that RNF181 depletion could inhibit cell proliferation speed in both BT549 and MDAMB231 cells (Fig. 2a, b). We further investigate the migration capacity in BT549 and MDAMB231 cells. The wound-healing assay shows that siRNF181 significantly inhibits the migration capability in both BT549 and MDAMB231 cells (Fig. 2c–f). Further trans-well assay shows that RNF181 knocking down decreases the number of migrated cells in BT549 and MDAMB231 cells (Fig. 2g, h).

**Fig. 2:** RNF181 promotes cell proliferation and migration in triple negative breast cancer cells. **a**, **b** Depletion of RNF181 inhibits the proliferation of triple negative breast cancer cells. BT549 and MDA-MA-231 were transfected with siControl or siRNF181. There were two different siRNA be used. After 24 h, the assay was CCK8 used to determine the cellar metabolic activity at indicated time points after infection. Experiments were done in triplicates. *P < 0.05; **P < 0.01; ***P < 0.001 for cell growth comparison. **c**–**f** Wound-healing assay of BT549 and MDA-MB-231 cells were transfected with siControl or siRNF181. Quantification of wound closure at the indicated time points. Data are presented as ± SD. **, P < 0.01, ***, P < 0.001. **g**, **h** RNF181 depletion inhibits TNBC cell migration in BT549 and MDA-MB-231 cells. Two independent siRNA were used in the study. Transwell was used to check the migration capacity. The cell number was counted and data are presented as ± SD. **, P < 0.01, ***, P < 0.001

### RNF181 facilitates Hippo/YAP signaling in TNBC cells

We further investigated the role of RNF181 in Hippo/YAP signaling. RNF181 depletion significantly decreased YAP protein level via two independent siRNAs in BT549 and MDAMB231 cells (Fig. 3a, b). We further investigate Hippo signaling activity via TEAD-luciferase activity. Luciferase assay showed that RNF181 depletion decreased TEAD luciferase activity in both BT549 and MDAMB231 cells (Fig. 3c, d). Besides, we measured the Hippo/YAP target genes in both of the two cells lines. QPCR assay showed that RNF181 depletion decreased Hippo/YAP target gene expression in MDAMB231 and BT549 cells (CTGF and CYR61) (Fig. 3e, f).

**Fig. 3:** RNF181 promotes Hippo signaling in triple negative breast cancer cells. **a** RNF181 consumption decreased YAP protein levels in BT549 cells. BT549 cells were transfected with siControl or siRNF181. After 48 h, cells were harvested for western blot analysis. RNF181 and YAP protein levels were determined by Western blot. Actin was used as internal control. **b** RNF181 consumption decreased YAP protein levels in MDAMB231 cells. MDAMB231 cells were transfected with siControl or siRNF181. After 48 h, cells were harvested for western blot analysis. RNF181 and YAP protein levels were determined by Western blot. Actin was used as internal control. **c** RNF181 depletion decreased TEAD Luciferase activity in BT549 cells. BT549 cells were transfected with siControl or siRNF181. After 24 h, cells were transfected with TEAD luciferase reporter plasmids. After 24 h, cells harvested for luciferase activity analysis. **d** RNF181 depletion decreased TEAD Luciferase activity in MDAMB231 cells. MDAMB231 cells were transfected with siControl or siRNF181. After 24 h, cells were transfected with TEAD luciferase reporter plasmids. After 24 h, cells harvested for luciferase activity analysis. **e** RNF181 consumption decreased YAP target gene expression in BT549 cells. BT549 cells were transfected with siControl or siRNF181. After 48 h, total RNA was extracted for gene expression analysis. *P < 0.05; ** P < 0.01; ***P < 0.001 for target gene expression comparison. **f** RNF181 consumption decreased YAP target gene expression in MDAMB231 cells MDAMB231 cells were transfected with siControl or siRNF181. After 48 h, total RNA was extracted for gene expression analysis. *P < 0.05; ** P < 0.01; ***P < 0.001 for target gene expression comparison

### RNF181 promotes migration and invasion via activating Hippo/YAP signaling in TBNC cells

We further investigated the logic link between cancer phenotype and Hippo signaling in TNBC cells. In Fig. 4a, decreased YAP protein level could be rescued by further YAP overexpression. The cell migration assay showed that RNF181 could inhibit cell migration in TNBC, which effect could be rescued by YAP overexpression in BT549 cells and MDAMB231 cells (Fig. 4b–e). Besides YAP overexpression could also rescued the invasion capacity, which was caused by RNF181 knocking down in BT549 and MDAMB231 cells (Fig. 4f, g).

**Fig. 4:** RNF181 promotes cancer cell migration and invasion through Hippo/YAP signaling. **a** RNF181 consumption decreased YAP protein level, which effect could be reversed by YAP over-expressed. BT549 cells were transfected with siControl or siRNF181. After 24 h, cells were transfected with Myc-YAP or Myc. After 48 h, cells were harvested for western blot analysis. RNF181 and YAP protein levels were determined by Western blot. Actin was used as internal control. **b**, **c** Wound-healing assay indicated that RNF181 consumption decreased BT549 cell migration capacity, which effect could be reversed by YAP over-expressed. BT549 cells were transfected with siControl or siRNF181. After 24 h, cells were transfected with Myc-YAP or Myc. Quantification of wound closure at the indicated time points. Data are presented as ± SD. **, P < 0.01, ***, P < 0.001 (student’s t-test). **d**, **e** Wound-healing assay indicated that RNF181 consumption decreased MDAMB231 cell migration capacity, which effect could be reversed by YAP over-expressed. MDAMB231 cells were transfected with siControl or siRNF181. After 24 h, cells were transfected with Myc-YAP or Myc. Quantification of wound closure at the indicated time points. Data are presented as ± SD. **, P < 0.01, ***, P < 0.001 (student’s t-test). **f**, **g** RNF181 consumption decreased TNBC cell invasion capacity, which effect could be reversed by YAP over-expressed. BT549 cells were transfected with siControl or siRNF187. After 24 h, cells were transfected with Myc-YAP or Myc. After another 24 h, cancer cells were seeded into the chamber for trans-well assay. The cell number was counted and Data are presented as ± SD. **, P < 0.01, ***, P < 0.001 (student’s t-test)

### RNF181 stabilizes YAP protein and inhibits YAP protein poly-ubiquitination

We further carried out the immuno-staining of YAP and RNF181 in MDAMB231 cells. The immuno-staining showed that both YAP and RNF181 localized in the nuclear (Fig. 5a). The immuno-precipitation showed that RNF181 could associate with YAP in the MDAMB231 cells (Fig. 5b). We analyzed the half-life of YAP protein with or without RNF181. The protein half-life assay showed that RNF181 depletion significantly decreased the YAP protein stability (Fig. 5c, d). Also, RNF181 associated with phospho-YAP (S127) protein in BT549 cells (Fig. 5e). The protein half-life assay showed that RNF181 depletion significantly decreased the phospho-YAP (S127) protein stability (Fig. 5f, g). Besides, YAP protein decrease by RNF181 knocking-down was diminished by the proteasome inhibitor treatment (Fig. 6a). Further ubiquitin-based immuno-precipitation assay showed that the existence of RNF181 could decrease the K48-linked ubiquitination of YAP in HEK293 cells (Fig. 6b).

**Fig. 5:** RNF181 facilitates YAP protein stability and inhibits YAP K48-linked poly-ubiquitination. **a** Intracellular localization analysis of RNF181 and YAP by immunofluorescence assay. BT549 cells were cultured in normal medium before fixation. Intracellular localization of YAP (red) and RNF181 (green) were shown. Nuclei (blue) were stained with 4′,6-diamidino-2-phenylindole (DAPI). **b** Co-IP assay revealed association between endogenous RNF181 and YAP protein in HEK293T cells. HEK293T cells were harvested with RIPA lysis buffer. CO-IP was performed using antibody as indicated. **c**, **d** RNF181 consumption decreased YAP half-life in BT549 cells. BT549 cells were transfected with 50 µM siControl or siRNF181. After 24 h, cells were treated with 100 µM cycloheximide/vehicle for indicated times. Cell lysates were prepared for Western blot analysis. The results are representative for three independent experiments. The YAP relative density was measured by Image J software. **e** Co-IP assay revealed association between endogenous RNF181 and phospho-YAP (S127) protein in BT549 cells. BT549 cells were harvested with RIPA lysis buffer. CO-IP was performed using antibody as indicated. **f**, **g** RNF181 consumption decreased phospho-YAP (S127) half-life in BT549 cells. BT549 cells were transfected with 50 µM siControl or siRNF181. After 24 h, cells were treated with 100 µM cycloheximide/vehicle for indicated times. Cell lysates were prepared for Western blot analysis. The results are representative for three independent experiments. The phospho-YAP (S127) relative density was measured by Image J software

**Fig. 6:** The hypothesis model of RNF181 regulating Hippo signal in triple negative breast cancer. **a** In the presence of the proteasome inhibitor MG132, the degradation effect of RNF181 on YAP did not further decrease YAP protein levels. BT549 cells were transfected with siRNF181 or siControl. After 24 h, cells were treated with 10 µM MG132/vehicle for 6 h. Cell lysates were prepared for Western blot analysis. The results are representative for three independent experiments. **b** RNF181 decreased K48-linked poly-ubiquitination of YAP. HEK293T cells were transfected with 0.5 µg Flag-RNF181 or Flag vector, together with 1 µg HA-K48 Ubi and Myc-YAP plasmid. The cell extracts were immunoprecipitated with HA antibody. The K48 specific poly-ubiquitinated YAP was detected via western blotting analysis. **c** RNF181 protein is related to YAP, which promotes YAP target gene transcription by promoting YAP stability and inhibits YAP degradation by inducing YAP K48 linked polyubiquitination

## Discussion

In our current study, we investigate the role of RNF181 in modulating TNBC cancer cell progression. RNF181 is found to associate with YAP and promoted YAP protein stability and Hippo signaling activation via inhibiting K48-linked poly-ubiquitination (Fig. 6). Besides, RNF181 is elevated in breast cancer, compared with normal breast tissue, while both RNF181 and YAP are correlated with poor prognosis in TNBC. Our study provided a novel insight into the post-translational mechanism in YAP/Hippo signaling. RNF181 could be an interesting marker for TNBC therapeutics and diagnostics.

Numbers of studies showed that the Hippo/YAP signaling play important role in carcinogenesis in several human cancer [20]. For example, YAP constitutive activation could lead to live cancer and lung cancer in mice models [21, 22]. Besides, YAP was shown to mediate several cancer related phenotypes, including migration, invasion, anti-apoptosis and epithelial–mesenchymal transition (EMT) [23]. When it comes to the TNBC, the dys-regulation of Hippo/YAP axis was found in TNBC tumors, such as YAP gene amplification and FAT mutations. Besides, YAP expression level was found to correlate with poor survival and progression stage in TNBC patients [24, 25]. YAP protein depletion could inhibit TNBC cell growth and invasion capacity in vivo and in vitro [26]. Since YAP is so critical in TNBC, it could be a promising strategy to target YAP for TNBC.

YAP protein contains three domains, including transcriptional activation domain, WW domain and TEAD interaction domain [10]. The WW domain modulates YAP subcellular localization, while TEAD interaction domain is responsible to interact with other transcriptional factors, such as TEAD and RUNX [27, 28]. YAP protein is the key mediator for the activation of Hippo signaling and subject to several translational modifications, such as phosphorylation and ubiquitination. For example, YAP could be phosphorylated in multiple sites by several kinases, which subsequently lead to the YAP cytoplasmic retention and YAP protein degradation [29, 30]. Besides, YAP protein also subject to ubiquitin modification. For example, FBW7, one E3 ubiquitin ligase could promote YAP protein K48-linked ubiquitination and degradation [31, 32]. Also SCF E3 ubiquitin ligases complex could also associate with YAP and promote YAP protein degradation [33]. In our current study, we observed that RNF181 could stabilize YAP protein and inhibit K48-linked ubiquitination and degradation. This finding could provide an unconventional regulation mechanism in controlling Hippo/YAP signaling by non-degradation ubiquitination manner.

RNF181 belongs to the RING family E3 ligase family, while the RING domain is responsible for the E3 ligation function. RNF181 is required for several physiological functions. For example, RNF181 is important to modulate integrin function in platelet [16]. In cancers, RNF181 was found to be elevated in several human malignancies. RNF181 could interact with CARD11 and promote NFKB signaling in lymphoma cells [17]. Besides, RNF181 was shown to promote colon cancer viability and angiogenesis [34]. Here, our results indicate that RNF181 could promote cell migration and proliferation in TNBC via activating Hippo/YAP signaling. Besides, we also showed that RNF181 was increased in breast cancer. This could indicate that RNF181 could stabilize YAP protein via a non-proteolytic manner, which could provide novel insight in the role of ubiquitin modification in YAP protein and Hippo signaling.

## Conclusion

We identified an interesting E3 ligase RNF181 in facilitating Hippo/YAP signaling in TNBC cells. RNF181 could promote TNBC cell invasion and proliferation via stabilizing YAP protein. As a novel modulator of Hippo signaling, disturbing RNF181 activity or affecting RNF181 expression could be a plausible way to overcome YAP-driven breast cancer among TNBC patients.

## Abbreviations

TNBC: Triple negative breast cancer
YAP: Yes-associated protein
TEAD: TEA domain transcriptional factor
RING: Really interesting new gene
RNF181: RING finger protein 181
ER: Estrogen receptor
LATS: Large tumor suppressor kinase

## References

[1] Bianchini G, Balko JM, Mayer IA, Sanders ME, Gianni L (2016). Triple-negative breast cancer: challenges and opportunities of a heterogeneous disease. Nat Rev Clin Oncol.

[2] Collignon J, Lousberg L, Schroeder H, Jerusalem G (2016). Triple-negative breast cancer: treatment challenges and solutions. Breast Cancer.

[3] Shah SP (2012). The clonal and mutational evolution spectrum of primary triple-negative breast cancers. Nature.

[4] Hayashi S, Yokoyama H, Tamura K (2015). Roles of Hippo signaling pathway in size control of organ regeneration. Dev Growth Differ.

[5] Meng Z, Moroishi T, Guan KL (2016). Mechanisms of Hippo pathway regulation. Genes Dev.

[6] Santucci M (2015). The Hippo pathway and YAP/TAZ-TEAD protein-protein interaction as targets for regenerative medicine and cancer treatment. J Med Chem.

[7] Harvey KF, Zhang X, Thomas DM (2013). The Hippo pathway and human cancer. Nat Rev Cancer.

[8] Pan D (2010). The hippo signaling pathway in development and cancer. Dev Cell.

[9] Wang L (2019). Unbalanced YAP-SOX9 circuit drives stemness and malignant progression in esophageal squamous cell carcinoma. Oncogene.

[10] Sudol M, Shields DC, Farooq A (2012). Structures of YAP protein domains reveal promising targets for development of new cancer drugs. Semin Cell Dev Biol.

[11] Overholtzer M (2006). Transforming properties of YAP, a candidate oncogene on the chromosome 11q22 amplicon. Proc Natl Acad Sci USA.

[12] Zhang K (2015). YAP and TAZ take center stage in cancer. Biochemistry.

[13] Zanconato F (2015). Genome-wide association between YAP/TAZ/TEAD and AP-1 at enhancers drives oncogenic growth. Nat Cell Biol.

[14] Li Z (2010). Structural insights into the YAP and TEAD complex. Genes Dev.

[15] Brophy TM (2008). RN181, a novel ubiquitin E3 ligase that interacts with the KVGFFKR motif of platelet integrin alpha(IIb)beta3. Biochem Biophys Res Commun.

[16] Raab M (2010). Protein interactions with the platelet integrin alpha(IIb) regulatory motif. Proteomics.

[17] Pedersen SM, Chan W, Jattani RP, Mackie DS, Pomerantz JL (2015). Negative regulation of CARD11 signaling and lymphoma cell survival by the E3 ubiquitin ligase RNF181. Mol Cell Biol.

[18] Xue M (2019). Regulation of estrogen signaling and breast cancer proliferation by an ubiquitin ligase TRIM56. Oncogenesis.

[19] Yang H (2018). SMURF1 facilitates estrogen receptor a signaling in breast cancer cells. J Exp Clin Cancer Res CR.

[20] Zanconato F, Cordenonsi M, Piccolo S (2016). YAP/TAZ at the roots of cancer. Cancer Cell.

[21] Zhang W (2015). YAP promotes malignant progression of Lkb1-deficient lung adenocarcinoma through downstream regulation of survivin. Cancer Res.

[22] Perra A (2014). YAP activation is an early event and a potential therapeutic target in liver cancer development. J Hepatol.

[23] Nguyen CDK, Yi C (2019). YAP/TAZ signaling and resistance to cancer therapy. Trends Cancer.

[24] Liu CH, Chang C, Sy E, Lai HW, Kuo YL (2015). Metaplastic breast carcinoma with multiple muscle metastasis: a case report. Medicine.

[25] Vici P (2016). Topographic expression of the Hippo transducers TAZ and YAP in triple-negative breast cancer treated with neoadjuvant chemotherapy. J Exp Clin Cancer Res CR.

[26] Sorrentino G (2017). Glucocorticoid receptor signalling activates YAP in breast cancer. Nat Commun.

[27] Zhang L (2008). The TEAD/TEF family of transcription factor Scalloped mediates Hippo signaling in organ size control. Dev Cell.

[28] Zhao B (2008). TEAD mediates YAP-dependent gene induction and growth control. Genes Dev.

[29] Cho YS (2018). Regulation of Yki/Yap subcellular localization and Hpo signaling by a nuclear kinase PRP4K. Nat Commun.

[30] Huang J, Wu S, Barrera J, Matthews K, Pan D (2005). The Hippo signaling pathway coordinately regulates cell proliferation and apoptosis by inactivating Yorkie, the Drosophila Homolog of YAP. Cell.

[31] Zhang Q (2016). Fbxw7 deletion accelerates Kras(G12D)-driven pancreatic tumorigenesis via yap accumulation. Neoplasia.

[32] Tu K (2014). Fbxw7 is an independent prognostic marker and induces apoptosis and growth arrest by regulating YAP abundance in hepatocellular carcinoma. Mol Cancer.

[33] Zhao B, Li L, Tumaneng K, Wang CY, Guan KL (2010). A coordinated phosphorylation by Lats and CK1 regulates YAP stability through SCF(beta-TRCP). Genes Dev.

[34] Gupta A (2015). Abrogation of AuroraA-TPX2 by novel natural inhibitors: molecular dynamics-based mechanistic analysis. Jc Receptor Signal Trans Res.

